# Protective Effects of Curcumin-Regulated Intestinal Epithelial Autophagy on Inflammatory Bowel Disease in Mice

**DOI:** 10.1155/2022/2163931

**Published:** 2022-04-29

**Authors:** Jianhua Hong

**Affiliations:** Department of Digestive Internal Medicine, Tonglu First people's Hospital, Tonglu, Hangzhou 311500, China

## Abstract

**Objective:**

This study was aimed at exploring the ameliorating effect of curcumin (Cur) on inflammatory bowel disease (IBD) in mice induced by 3% dextran sodium sulfate (DSS) by regulating intestinal epithelial cell autophagy.

**Methods:**

45 BALB/c mice were randomly divided into three groups: control group, DSS group, and Cur group, with 15 mice in each group. Expect for the control group, 3% DSS was freely drunk by the mice for 7 days to induce acute IBD, and the Cur group was given Cur gavage treatment. Hematoxylin-Eosin (HE) staining was performed to observe the pathological changes of mice colon tissue. The formation of autophagosomes in intestinal epithelial cells was detected by transmission electron microscopy (TEM). The protein expressions of LC3-II/LC3-I, p62, and Beclin1 were detected by Western blot.

**Results:**

Compared with that of the control group, body weight of mice in DSS group was significantly reduced, stool was not formed or presented with loose stools, there was occult blood or blood in the stool, hair color lost luster, disease activity index (DAI) score was significantly increased, and colonic mucosal epithelial cells showed colitis; LC3-II/LC3-I and Beclin1 expression were significantly decreased (*P* < 0.05), p62 was significantly increased, and autophagy was not obvious. In addition, compared with that of the DSS group, the diet of mice in the Cur group was improved, the decline of body weight was slowed down, the hair glossiness was restored, the blood in the stool gradually decreased or occulted, the DAI score was decreased, the colon tissue was significantly improved, the expressions of LC3-II/LC3-I and Beclin1 were significantly increased (*P* < 0.05), and the p62 was significantly decreased.

**Conclusions:**

The effect of Cur on IBD mice was related to the regulation of the expression of autophagy pathway proteins LC3-II/LC3-I, Beclin1, and p62 in intestinal epithelial cells.

## 1. Introduction

Inflammatory bowel disease (IBD) is a special nonspecific chronic disease, mainly including Crohn's disease (CD) and ulcerative colitis (UC) [1]. UC is an immune disease characterized by inflammation confined to the colonic mucosa and submucosa, accompanied by significant intestinal immune imbalance [2]. At present, the drugs for the treatment of UC mainly contain salicylic acid preparations, and the research and development of new biological preparations are also ongoing. However, the long-term use of traditional medicines leads to poor patient compliance, and it is better to research and develop new medicines with fewer side effects. Most patients in China need to take long-term medication, which is under great economic pressure and has a wide range of promotion [3]. Therefore, it is of certain clinical significance to find traditional Chinese medicines (TCM) with high cost performance, good curative effect, and less toxic and side effects to treat IBD. Curcumin (Cur) is a chemical component extracted from the rhizomes of plants such as Zingiberaceae and Araceae. It is a pigment with few diketones in the plant kingdom and is a diketone compound. It is characterized by an orange-yellow crystalline powder with a slightly bitter taste [4]. The role of Cur in the treatment of IBD has been confirmed in clinical reports, but the specific mechanism is still unclear. It has been reported that Cur can improve IBD in mice by inhibiting the STAT3 signaling pathway in intestinal epithelial cells, relieve ulcerative colitis by regulating the expression of P38MAPK in colon tissue, and relieve inflammation by regulating intestinal flora [5]. However, there is no relevant report on the effect of Cur on intestinal immunity. Intestinal epithelial cells are located in the basal layer of intestinal epithelial cells and play an important role in maintaining intestinal homeostasis. Autophagy of intestinal epithelial cells is one of the important safeguard factors for intestinal epithelial cell homeostasis and intestinal mucosal barrier integrity and is involved in intestinal immune regulation and pathogen clearance [6]. Beclin1 is an important switch for initiating autophagy and regulates autophagy-related genes by forming a complex with type III PI3K. Ubiquitin-binding protein-1 (p62) is an autophagy substrate protein [7].

When autophagy occurs, p62 binds to ubiquitin-related proteins in the cytoplasm to form a complex with LC3, which is mediated by LC3 into autophagosomes, and finally completes degradation in autophagosomes. At present, commonly used autophagy detection methods such as LC3-II/LC3 and observation of autophagosome morphology under a transmission electron microscope (TEM) have been widely used in the basic research of autophagy [8]. In the pathological process of IBD, the intestinal epithelial barrier is destroyed and the permeability of the intestinal mucosa is increased, which leads to the swelling of intestinal epithelial cells and nutritional deficiency. The swelling of intestinal epithelial cells has an inhibitory effect on autophagy [9]. Cur is an active ingredient extracted from the ginger plant turmeric. It was found that Cur can act on human monocytes and has the effect of inhibiting the production of the inflammatory mediator interleukin-1*β* (IL-1*β*), which was reflected by the great reduction of proportion of subgroups and obvious increase in activation of CD4+ T cells and CD8+ T cells [10]. In addition, the subpopulation and function of small intestinal epithelial cells are also significantly altered in a mouse model of acute ischemia-reperfusion (IR). Likewise, a hyperactivated state of gut innate immunity has also been found in samples from patients with intestinal IR [11, 12]. Studies have shown that dysfunction and subpopulation of intestinal epithelial cells are significantly associated with the severity of colonic inflammation. Cur has anti-inflammatory effects in the treatment of IBD [13]. However, the mechanism by which Cur participates in the repair of inflammatory damage in the body is unclear. Therefore, based on the establishment of a stable IBD model, the protective effect of Cur on damaged intestinal mucosa was explained in this work to explore its possible mechanism from autophagy and autophagy-related pathway proteins.

## 2. Materials and Methods

### 2.1. Experimental Animals

A total of 45 Specified Pathogen Free (SPF) BALB/c healthy male mice aged 6 to 8 weeks with body weight of 22 ± 2 g were purchased from Shanghai Sippr-BK laboratory animal Co. Ltd., China. This research complied with the *Regulations on the Management of Laboratory Animals* promulgated by the National Science and Technology Commission and the *Detailed Rules for the Management of Laboratory Animals* promulgated by the State Medical Administration, and all the contents involved met the requirements of the ethics committee of the hospital.

### 2.2. Experimental Main Drugs

Dextran sodium sulfate (DSS) was purchased from Sigma Company, USA; and Cur (PHLC ≥ 98%) was purchased from Nanjing Zelang Medical Technology Co., Ltd., China.

### 2.3. Modeling, Grouping, and Administration

45 BALB/c mice were randomly divided into 3 groups (blank control group, DSS group, and Cur group), with 15 mice in each group. The blank control group was given a free-drinking diet (other experimental procedures were the same as those in DSS group and the Cur group), and both the DSS group and the Cur group were given 3% DSS free drinking for 7 days to induce acute IBD. The shape of the feces of the mice was observed, and the fences were collected to detect occulting blood. In addition, the hair and mental state of mice were observed. In addition to repeating the experimental steps at the same time period every day, the DSS fluid should be ensured without interruptions. Until the 7th day, the model was successful if the mice did not suffer from listlessness, significant weight loss, loss of appetite, loss of hair luster, and obvious bloody stools.

Mice in the Cur treatment group were given Cur by garaging at 200 mg/kg on the 3rd day before modeling, with 3 times a day, while mice in the blank control group were garaged with an equal volume of normal saline for 7 consecutive days. During this period, the body weight of the mice was monitored and recorded every day, and mouse feces were collected for diarrhea index and stool blood index scoring.

### 2.4. Detected Indicators

After experiment (7 days after the administration), the fence characteristics and blood in stool, activity, spirit, diet, and body weight of mice were observed, and the DAI of mice was calculated to judge the modeling situation and observe the curative effect. DAI was the sum of the scores of body weight decline, stool characteristics, and blood in the stool. The scoring standards were as follows. No decline in body weight, decline > 1%~5%, decline > 5% ~10%, decline > 10% ~15%, and decline > 15% were counted as 0, 1, 2, 3, and 4 points, respectively; stool characteristics were normal, loose (mushy or semiformed stool, not adhering to the anus), and loose stool (watery stool) were counted as 0, 2, and 4 points, respectively; and no blood in the stool, fecal occult blood (+), and gross blood in the stool were counted as 0, 2, and 4 points, respectively. The DAI scoring of each mouse was the average of 3 detected results.

### 2.5. Colon Tissue Specimen

After the animal model was established, the mice were anesthetized, killed by neck breaking method, and the colorectal part between the cecum and anus was taken and the length of the colorectum was measured. A 1 cm section of the intestine was cut from the same part of the colorectum of each mouse and fixed in 4% paraformaldehyde solution for HE staining. The remaining intestinal tissues were used for observations under TEM and Western blot.

### 2.6. HE Staining

The main process of tissue HE staining [14] was described as follows. Colonic tissue was taken, fixed, embedded in paraffin, and sectioned at an interval of 4 *μ*m. After routine dewaxing, the slices were placed in hematoxylin aqueous solution and stained for 10 min. The slices were separated in acid water and ammonia water for a few seconds. Then, the slices were rinsed with water for 1 h and put into distilled water for a while. The slices were immersed in 70% and 90% alcohol and dehydrated for 10 min each. The stained slices were dehydrated with pure alcohol and then cleared with xylene. Gum was dropped on the transparent sections, which were coved with cover glass and fixed; after the gum was dry, it can be used for observation. Histological evaluation was graded from 0 to 5.

1. Level 0: normal form
2. Level 1: epithelial edema and partially separated apical cells
3. Level 2: ascend from the hinted villi cells
4. Level 3: lift cells from the top and sides (including surface villi crypts)
5. Level 4: partial necrosis of the lamina propria mucosa
6. Level 5: full-thickness mucosal necrosis

### 2.7. TEM to Detect Autophagy

TEM was adopted to detect the autophagy, and the specific steps were summarized as follows [15]. An appropriate amount of colon tissue was taken and fixed in 2.5% glutaraldehyde phosphate buffer for fixation. After overnight, colon tissue was rinsed with Phosphate-Buffered Saline (PBS) and fixed with 1% osmium acid. Then, the colon tissue was rinsed with PBS and stained in 2% uranyl acetate aqueous solution, dehydrated in different concentrations of ethanol gradient and 100% acetone, mixed and infiltrated in anhydrous acetone and embedded agent in a 1 : 1 volume, and then shaken for 2 h. Finally, the colon tissue was placed in an oven for polymerization at 37°C for 24 h, 45°C for 24 h, and 60°C for 48 h, repaired and sliced (about 120 nm), dyed, stained with 4% uranium acetate for 20 min, and stained with lead citrate for 5 min. After staining, it was placed on a single hole copper net, observed, recorded, and photographed under a TEM.

### 2.8. The Protein Expressions of LC3-II/LC3-in, p62, and Beclin1 Detected by Western Blot

The relative expression level of the target protein was detected by Western blot technology [16]. The protein samples were prepared with radioimmunoprecipitation assay (RIPA) high-efficiency lysate and phenylmethanesulfonyl fluoride (PMSF); the protein concentration was detected with bicinchoninic acid (BCA) kit. The protein was subjected to sodium dodecyl sulfate polyacrylamide gel electrophoresis (SDS-PAGE) gel electrophoresis, membrane transfer, sealing, specific binding with antibody, chemiluminescence development, photography, and preservation. In addition, the gray value of the strips was measured with Quantity One image.

### 2.9. Statistical Method

All data were analyzed by SPSS 20.0 statistical software, and the experimental data were expressed as $\bar{x}\pm s$. One-way analysis of variance was used to compare the mean values among multiple samples, and *P* < 0.05 indicated that the difference was statistically significant.

## 3. Results

### 3.1. The Effect of Cur on IBD in Mice

The diet, activity, hair color, and fence characteristics of mice in the control group were normal, and body weight did not fluctuate significantly, as shown in Figure 1(a). After modeling, mice in the DSS group gradually showed anorexia, less activity, and significantly reduced body weight, unformed stools or loose stools, occult blood in stools or blood in the stool, loss of hair color, and a significant increase in DAI score (*P* < 0.05), as shown in Figure 1(e). After medication intervention in the Cur group, compared with the DSS group, the diet situation was improved, the decline in body weight slowed down, the gloss of the hair was restored, the blood in the stool gradually decreased or occulted, and the DAI score decreased (*P* < 0.05). Further significance analysis of the diarrhea index score and stool blood index score of mice showed that the diarrhea index and stool blood index scoring of mice in the Cur group were lower than those in the DSS group (*P* < 0.05), as shown in Figures 1(b) and 1(c).

In addition, paraffin section of mice colons was performed for HE staining and pathological scoring of staining results, as shown in Figure 1(d). The results showed that the colonic mucosa of mice in blank control group had a complete structure without inflammatory cell infiltration, with clear outline and continuous intestinal epithelium. The intestinal epithelial cells and glands were arranged neatly, and the subcellular matrix and blood vessels were normal. In the DSS group, colonic mucosal epithelial cells were widely missing, most of the glands were incomplete, and inflammatory cells were extensively infiltrated and presenting in colitis. The colonic mucosal glands in the Cur group were basically intact, with a small amount of inflammatory cell infiltration or crypt destruction in the local area, which was significantly improved compared with the DSS group.

### 3.2. The Effect of Cur on Autophagy of Mouse Intestinal Epithelial Cells

Compared with the control group, the autophagy of intestinal epithelial cells of mice in the DSS group was significantly reduced, and the formation of vacuolar structures of bilayer was less observed under the microscope, while the autophagy of intestinal epithelial cells in the Cur group was significantly increased, and more vacuolar structures of bilayer were observed under the microscope, containing cytoplasmic components such as mitochondria, as shown in Figure 2.

### 3.3. Results of Western Blot

Compared with the control group, the expressions of LC3-II/LC3-I and Beclin1 in the DSS group were significantly reduced (*P* < 0.05), while the expression of p62 was significantly increased (*P* < 0.05). Compared with the DSS group, the expressions of LC3-II/LC3-I and Beclin1 in the Cur group were significantly increased (*P* < 0.05), and the expression of p62 was decreased (*P* < 0.05), as shown in Figure 3.

## 4. Discussion

The main clinical symptoms of UC are diarrhea, abdominal pain, and tenesmus with blood in the stool. At present, the specific etiology of UC has not been elucidated in detail, but many pathological examinations and experimental models have proved that abnormal expression of the immune system is an important factor causing intestinal inflammation and tissue damage [17]. At present, UC is difficult to treat, has a long course of disease, and is easy to cause cancer. Therefore, it has been recognized as one of the most intractable diseases in the world. Traditional drugs for the treatment of UC show large side effects after long-term use and are quite expensive compared with biological preparations developed in recent years, which is not conducive to widespread clinical application. Therefore, it is of great significance to find affordable drugs with less adverse reactions [18]. Based on the important role of intestinal epithelial cells in intestinal inflammation and the ability of Cur to alleviate related inflammation, a novel mechanism was established in this work to investigate the effect of Cur on a subgroup of intestinal epithelial cells in DSS ulcerative colitis mice. The data have confirmed that various factors such as environment, genetics, and immunity are closely related to the occurrence and development of IBD, especially the abnormal autophagy of cells in the body [19]. Studies have shown that Cur may inhibit the DSS-induced IBD process and alleviate the disease by reducing the inflammatory response and the expression of autophagy-related factors [20]. In this work, Cur was used to treat intestinal epithelial cells of mouse colon tissue and the changes in the expression levels of autophagy-related factors in the cells were measured to further clarify the mechanism of Cur alleviating IBD.

The PI3K/Akt/mTOR signaling pathway participates in and regulates autophagy in the body [21]. p62 can directly bind to the autophagy marker protein LC3, so it is the preferred target for examining autophagy. In the process of IBD, the pathological features show the breakdown of the intestinal epithelial cell barrier and the increase in the permeability of the intestinal mucosa, which leads to the swelling of the intestinal epithelial cells and nutritional deficiency, but the swelling of the intestinal epithelial cells can effectively inhibit the phagocytosis level [22]. In the process of autophagy formation, LC3-I can bind to phosphatidylethanolamine (Kepha-lin) and form LC3-II, so the conversion of LC3-I to LC3-II is an important marker of autophagosome formation [23]. Studies have confirmed that the expression of autophagy signature protein p62 is negatively correlated with the level of autophagy [24]. Therefore, the ratio of LC3-II/LC3-I and the degradation of p62 protein were detected and analyzed in this work to reflect the changes in the autophagy level of intestinal epithelial cells in mouse colon tissue after Cur treatment.

The results showed that compared with the control group, autophagy in intestinal epithelial cells of DSS group was significantly decreased, LC3-II/LC3-I and Beclin1 expression were significantly decreased, and p62 was significantly increased. Such results indicated that autophagy was involved in colon tissue of IBD mice, inhibiting the level of autophagy. The expressions of LC3-II/LC3-in and Beclin1 were significantly increased in the Cur group, while the expression of p62 was significantly decreased, indicating that Cur can improve the level of autophagy. The process of autophagy is mainly divided into activation under stress, formation and extension of separation membrane, and formation of autophagy-lysosome. Inflammation is the body's self-protective response caused by microbial pathogen infection or tissue damage, and inflammatory bowel disease is a chronic nonspecific inflammatory disease of the gut [25]. Autophagy can affect the process of inflammatory diseases through a variety of methods, such as the clearance of pathogens, the intervention of antigen presentation, and the regulation of inflammatory cytokine production [26]. Other studies have confirmed that the lack of autophagy can lead to the abnormality of intestinal microflora and the destruction of intestinal morphology, which eventually leads to the disturbance of intestinal function and the occurrence of pathological changes [27]. Therefore, Cur can increase the expression level of autophagy protein in IBD mice, which may be one of the molecular mechanisms for the treatment of IBD intestinal inflammation.

## Figures and Tables

**Figure 1:** Improvement of Cur on DSS-induced IBD in mice. (a) The changes in body weight of mice; (b) the diarrhea index scoring curve of mice; (c) the scoring curve of stool blood index of mice; (d) HE staining image of mice colon (A: blank control group; B: DSS group; C: Cur group, HE×200); (e) DAI scoring of mice in each group. ^∗^Compared with the control group, *P* < 0.05; ^#^compared with the DSS group, *P* < 0.05.

**Figure 2:** The effect of Cur on autophagy in intestinal epithelial cells of IBD mice (transmission electron microscope, ×6000).

**Figure 3:** The expression of each protein in the colon tissue. ^∗^Compared with the control group, *P* < 0.05; compared with the DSS group, *P* < 0.05.

## Data Availability

The data used to support the findings of this study are available from the corresponding author upon request.

## References

[1] Lucas C., Salesse L., Hoang M. (2020). Autophagy of intestinal epithelial cells inhibits colorectal carcinogenesis induced by colibactin-producing *Escherichia coli* in *Apc*^_Min/+_^ mice. *Gastroenterology*.

[2] Tang Y., Li F., Tan B. (2014). Enterotoxigenic *Escherichia coli* infection induces intestinal epithelial cell autophagy. *Veterinary Microbiology*.

[3] Chang C. J., Lin J. F., Hsiao C. Y. (2017). Lutein induces autophagy via Beclin-1 upregulation in IEC-6 rat intestinal epithelial cells. *American Journal of Chinese Medicine*.

[4] Liang C., Feng Z., Manthari R. K. (2020). Arsenic induces dysfunctional autophagy via dual regulation of mTOR pathway and Beclin1-Vps34/PI3K complex in MLTC-1 cells. *Journal of Hazardous Materials*.

[5] Masuda G., Yashiro M., Kitayama K. (2016). Clinicopathological correlations of autophagy-related proteins LC3, Beclin 1 and p62 in gastric cancer. *Anticancer Research*.

[6] Schmitz K. J., Ademi C., Bertram S., Schmid K. W., Baba H. A. (2016). Prognostic relevance of autophagy-related markers LC3, p62/sequestosome 1, Beclin-1 and ULK1 in colorectal cancer patients with respect to KRAS mutational status. *World Journal of Surgical Oncology*.

[7] Goulielmaki M., Koustas E., Moysidou E. (2016). BRAF associated autophagy exploitation: BRAF and autophagy inhibitors synergise to efficiently overcome resistance of BRAF mutant colorectal cancer cells. *Oncotarget*.

[8] Macias-Ceja D. C., Cosín-Roger J., Ortiz-Masiá D. (2017). Stimulation of autophagy prevents intestinal mucosal inflammation and ameliorates murine colitis. *British Journal of Pharmacology*.

[9] Xu-Tao L., Xiao-Bin Z., De-Jun F. (2018). MicroRNA-143 targets ATG2B to inhibit autophagy and increase inflammatory responses in Crohn's disease. *Inflammatory Bowel Diseases*.

[10] Lassen K. G., Xavier R. J. (2017). Genetic control of autophagy underlies pathogenesis of inflammatory bowel disease. *Mucosal Immunology*.

[11] Moriggi M., Pastorelli L., Torretta E. (2017). Contribution of extracellular matrix and signal mechanotransduction to epithelial cell damage in inflammatory bowel disease patients: a proteomic study. *Proteomics*.

[12] Liu S., Qian L., Zhang M. T. (2016). Curcumin ameliorates neuropathic pain by down-regulating spinal IL-1*β* via suppressing astroglial NALP1 inflammasome and JAK2-STAT3 signalling. *Scientific Reports*.

[13] Paulino N., Paulino A. S., Diniz S. N. (2016). Evaluation of the anti-inflammatory action of curcumin analog (DM1): effect on iNOS and COX-2 gene expression and autophagy pathways. *Bioorganic & Medicinal Chemistry*.

[14] Runz M., Rusche D., Schmidt S. (2021). Normalization of HE-stained histological images using cycle consistent generative adversarial networks. *Diagnostic Pathology*.

[15] Zhang Y., Liu D., Hu H., Zhang P., Xie R., Cui W. (2019). HIF-1*α*/BNIP3 signaling pathway-induced-autophagy plays protective role during myocardial ischemia-reperfusion injury. *Biomedicine & Pharmacotherapy*.

[16] Pillai-Kastoori L., Schutz-Geschwender A. R., Harford J. A. (2020). A systematic approach to quantitative Western blot analysis. *Analytical Biochemistry*.

[17] Ping G., Liu H., Huang H., Zhang Q., Strober W., Zhang F. (2017). The inflammatory bowel disease–associated autophagy gene Atg16L1T300A acts as a dominant negative variant in mice. *Journal of Immunology*.

[18] Yue W., Liu Y., Li X., Lv L., Huang J., Liu J. (2019). Curcumin ameliorates dextran sulfate sodium-induced colitis in mice via regulation of autophagy and intestinal immunity. *The Turkish Journal of Gastroenterology*.

[19] Li X., Feng K., Jiang L. (2017). Curcumin inhibits apoptosis of chondrocytes through activation ERK1/2 signaling pathways induced autophagy. *Nutrients*.

[20] Ming J., Zhu Y., Ding Z., Yanduo J., Guocheng J. (2019). Interleukin 7 receptor activates PI3K/Akt/mTOR signaling pathway via downregulation of Beclin-1 in lung cancer. *Molecular Carcinogenesis*.

[21] Lin Y., Huang S., Chen Y. (2020). Helix B surface peptide protects cardiomyocytes from hypoxia/reoxygenation-induced autophagy through the PI3K/Akt pathway. *Journal of Cardiovascular Pharmacology*.

[22] Wang S. L., Shao B. Z., Zhao S. B. (2019). Intestinal autophagy links psychosocial stress with gut microbiota to promote inflammatory bowel disease. *Cell Death & Disease*.

[23] Retnakumar S. V., Muller S. (2019). Pharmacological autophagy regulators as therapeutic agents for inflammatory bowel diseases. *Trends in Molecular Medicine*.

[24] Zaarour R. F., Azakir B., Hajam E. Y. (2021). Role of hypoxia-mediated autophagy in tumor cell death and survival. *Cancers (Basel)*.

[25] Dong J., Liang W., Wang T. (2019). Saponins regulate intestinal inflammation in colon cancer and IBD. *Pharmacological Research*.

[26] Haq S., Grondin J., Banskota S., Khan W. I. (2019). Autophagy: roles in intestinal mucosal homeostasis and inflammation. *Journal of Biomedical Science*.

[27] Cosin-Roger J., Simmen S., Melhem H. (2017). Hypoxia ameliorates intestinal inflammation through NLRP3/mTOR downregulation and autophagy activation. *Nature Communications*.

